# Efficacy and Safety of Electroacupuncture in the Treatment of Cerebral Infarction: Systematic Review and Meta-Analysis

**DOI:** 10.1155/2022/1350501

**Published:** 2022-06-28

**Authors:** Lan Xiang Wang, Wei Hong Li, Fang He

**Affiliations:** ^1^Department of Rehabilitation Medicine, The 8th Medical Center of Chinese PLA General Hospital, China; ^2^Beijing University of Chinese Medicine, China; ^3^Department of Outpatient, The 8th Medical Center of Chinese PLA General Hospital, China; ^4^Jia NO2 Niangniang Mansion, Xiangshan Road, Haidian District, Beijing 100093, China

## Abstract

**Purpose:**

The goal of this study was to see if electroacupuncture was effective and safe in the management of cerebral infarction. PubMed, Embase, Cochrane Library, and Web of Science were used to conduct a comprehensive literature survey.

**Methods:**

Basic features of 7 studies were identified using the searching strategy. The investigation was found in PubMed, Embase, and Web of Science, with the most recent search being in March 2022. “Electroacupuncture,” “cerebral infarction,” and their permutations were among the MeSH terms and free words used. As literature, two reviewers independently used a standardized form to gather pertinent data from qualifying research.

**Results:**

157 literatures were identified and evaluated. Electroacupuncture improved the BI score in individuals with cerebral infarction (mean difference = 0.10, 95 percent CI: 0.00-0.20, *p* = 0.04). Electroacupuncture enhanced BI score in individuals with cerebral infarction (mean difference = 0.10, 95 percent CI: 0.00-0.20, *p* = 0.04). The effects of electroacupuncture increased Fugl-Meyer index in patients with cerebral infarction (mean difference = 25.92, 95% CI: 25.28-26.56, *p* < 0.00001). Electroacupuncture effects decreased CSS in patients with cerebral infarction in the experiment group (mean difference = −2.10, 95% CI: -2.53–-1.67, *p* < 0.0001). Electroacupuncture also reduced CSS individuals with cerebral infarction in the control group; however, there was no statistically significant (risk difference = 0.06, 95 percent CI: 0.02-0.13, *p* = 0.12).

**Conclusion:**

This study demonstrated that electroacupuncture helped decreased CSS in patients with cerebral infarction.

## 1. Introduction

Acute cerebral infarction (ACEI) is a devastating cardiovascular and cerebrovascular disorder that affects millions of people every year [1].The death and disability rates are both extremely high [1]. The main cause of its pathogenesis is thrombosis or thrombus shedding on the arterial wall caused by atherosclerosis and multiple Takayasu arteritis, which flows into and blocks the cerebral artery through blood circulation, resulting in the disorder of brain blood supply and ischemic infarction in the dominated brain area [2]. The main clinical manifestations are as follows: weakness or numbness of one limb (with or without face); unclear speech or difficulty in understanding language; eyes staring to one side or vision loss, blurred; and sudden focal neurological deficits such as dizziness, vomiting, aphasia, disturbance of consciousness, or convulsions [3, 4]. Therefore, taking positive measures in the early stage of patients is the key to reduce death and disability. Individuals with an acute cerebral infarction are currently treated mostly by lowering intracranial pressure: dehydration, anti-infection, and controlling blood pressure [5]. The short-term effect is obvious, but there are many side effects and easy to relapse [6].

Traditional Chinese medicine classifies cerebral infarction, also known as ischemic stroke, as a type of stroke [7]. Wind, fire, phlegm, deficiency, and blood stasis are all common contributors to its occurrence [7]. Cerebral infarction is thought to be caused by a problem with the blood supply to the brain, as well as ischemia and hypoxia, according to modern medicine [8]. Ischemia and hypoxia will lead to brain tissue necrosis and softening and then lead to focal or complete neurological deficit. Cerebral infarction is characterized by quick commencement, a significant fatality rate, and a higher incidence of impairment [8]. At present, management of cerebral infarction is mainly through improving hemorheology, adjusting the balance of fibrinolytic system, and regulating blood lipid metabolism, body immunity, and neuron protection [8].

One of the most prevalent cerebrovascular illnesses seen in clinic is primary cerebral infarction, which seriously threatens the life of the elderly [9]. Poststroke depression (PSD) is a common complication of cerebral infarction patients [9]. The incidence rate of Dutch act is as high as 20%-60%. This has a negative impact on patients' prognosis and quality of life [9]. Some patients even have suicidal tendencies. Plasma homocysteine (HCY) and the presence of depression following a brain infarction are thought to be linked to the concentration of IL-1/tumor necrosis factor- (TNF-) *α* in the blood. Through detecting the plasma HCY level and serum IL-1*β* in depressed and nondepressed patients with primary cerebral infarction *β*, TNF-*α* is in correlation with the occurrence of depression in individuals that possess in individuals experiencing primary cerebral infarction depression, and the severity of depression is related to the initial cerebral infarction. The author will explore the level of plasma Hcy, and serum IL-1*β*/TNF-*α* level is used as a monitoring index of the severity of depression after primary cerebral infarction and to guide the feasibility of clinical treatment and prognosis of patients with primary cerebral infarction [10].

Acupuncture and moxibustion is a unique treatment method of traditional medicine in China, which has been applied for thousands of years [11]. Chinese electroacupuncture therapy believes that “from the situation of acupuncture acupoints and nerve segmentation, it seems that the essence of meridians may be a comprehensive functional system dominated by the nervous system, including nerves, body fluids, blood vessels and the time of controlling blood vessels” [12]. Some foreign scholars have shown that the mechanism of electroacupuncture may play a corresponding role by stimulating the nerves in the muscle [13, 14]. That is, electroacupuncture stimulates nerves to transmit signals to the notochord and brain to promote the release of neurotransmitters and neurohormones, so as to produce a certain therapeutic effect [15, 16]. The goal of this study was to see if electroacupuncture was effective and safe in the management of cerebral infarction.

## 2. Materials and Methods

### 2.1. Literature search

The investigation was found in PubMed, Embase, and Web of Science, with the most recent search being in March 2022. “Electroacupuncture,” “cerebral infarction,” and their permutations were among the MeSH terms and free words used. To locate new papers of interest, the reference lists of prior relevant reviews were manually searched. English or Chinese was the only languages allowed in the publications.

### 2.2. Inclusion and Exclusion Criteria

To determine which studies were eligible, the relevant inclusion criteria were used: (i) a cerebral infarction diagnosis was confirmed pathologically; (ii) the Barthel Index (BI), Fugl-Meyer index, Chinese Stroke Scale (CSS), and national institute of healthcare score (NIHSS) were evaluated in this study; and (iii) if multiple articles from the same patient cohort were found, the most comprehensive one was chosen. The following items were excluded from the study: (i) abstracts, reviews, case reports, or comment letters; (ii) animal research; (iii) duplicate publications; and (iv) articles that were not written in English or Chinese.

### 2.3. Data Extraction and Statistical Analysis

As literature, two reviewers independently used a standardized form to gather pertinent data from qualifying research [17]. Review Manager 5.3 was used to examine the data as literature [17]. The level of variability across research was investigated using a Chi-square based *Q* test, with *I*^2^ indicating the level of heterogeneity. Low heterogeneity was defined as *I*_250_ percent or *P* heterogeneity >0.1. *P* < 0.05 was considered as significant statistically.

## 3. Results

### 3.1. Features of Included Studies

This study was identified through systematic literature searching. 157 literatures were identified and evaluated.  Figure 1 depicts the book selection procedure.  Table 1 summarizes the main elements of seven research [18–24]. The number of people in the sample varied from 46 to 164.

### 3.2. Characteristics of Included Studies

The Cochrane Collaboration's technique for measuring risk of bias was used to assess the quality of the literatures (Figures 2(a) and 2(b)). Numerous studies were randomized, with proper allocation concealment procedures, insufficient outcome data, and double blinding (Figures 2(a) and 2(b)).

### 3.3. Electroacupuncture's Effects on Cerebral Infarction BI

The benefits of electroacupuncture on the BI rating of cerebral infarction were investigated in this study. Electroacupuncture enhanced BI score in individuals with cerebral infarction, as demonstrated in Figure 3(a) (mean difference = 0.10, 95 percent CI: 0.00-0.20, *p* = 0.04).

### 3.4. Electroacupuncture Effects on Fugl-Meyer Index of Cerebral Infarction

The present study analyzed the effects of electroacupuncture on Fugl-Meyer index of cerebral infarction. As shown in Figure 3(b), the effects of electroacupuncture increased Fugl-Meyer index in patients with cerebral infarction (mean difference = 25.92, 95% CI: 25.28-26.56, *p* < 0.00001).

### 3.5. Electroacupuncture's Effects on Cerebral Infarction CSS

The benefits of electroacupuncture on the CSS of cerebral infarction were investigated in this study. Electroacupuncture reduced CSS in individuals having cerebral infarction; although, the difference was not statically important after therapy (risk differential = 0.06, 95 percent CI: 0.02-0.13, *p* = 0.12).

### 3.6. The Effects of Electroacupuncture on NIHSS of Cerebral Infarction

The impacts of electroacupuncture on the NIHSS of cerebral infarction were investigated in this study. Electroacupuncture reduced NIHSS in individuals with cerebral infarction, as seen in Figure 3(d) (mean difference = -2.10, 95 percent CI: -2.53–-1.67, *p* < 0.00001).

### 3.7. Publication Bias

Funnel plots for meta-analysis of BI, Fugl-Meyer index, CSS, or NIHSS of cerebral infarction were shown in Figures 3–5. All of the funnel plots were symmetric, suggesting that there was no clear publishing bias.

## 4. Discussion

Cerebral infarction is a form of ischemic stroke that happens when the blood supply to the functioning part of the brain is cut off [25]. The blockage of blood supply leads to the injury and death of diseased tissues [26]. Cerebral infarction can lead to many results, such as loss of physiological function, paralysis, and even death [25]. Our findings revealed that 7 literatures with 854 participants were included in the meta-analysis, which was published between 2001 and 2020.

Acute cerebral infarction has always been a high incidence rate, high mortality, and disability rate [27]. Especially for the elderly, if we miss the early treatment, it is easy to cause sequelae such as disturbance of consciousness and hemiplegia. This will have a negative impact on one's standard of living and place a considerable financial strain on the household [28, 29]. Modern medicine believes that atherosclerosis is the pathological basis of acute cerebral infarction [29]. The increasing degree of atherosclerosis will form thrombus, block blood vessels, lead to complete occlusion of blood vessels, and cause ischemia, degeneration, and necrosis of nerve cells in brain tissue, resulting in corresponding symptoms of neurological deficit [30, 31]. The effects of electroacupuncture improved BI rating in participants with cerebral infarction (mean difference =0.10, 95 percent CI: 0.00-0.20, *p* = 0.04), according to the findings of a meta-analysis.

Electroacupuncture is to transmit stable and continuous electrical stimulation to acupoints through filiform needle [32]. Electrical stimulation parameters include frequency, intensity, time, and nature [33]. Numerous investigations have revealed that any change in one of the parameters will have different effects on the body [32, 33]. The present study showed that the effects of electroacupuncture increased Fugl-Meyer index in cerebral infarction patients.

Electroacupuncture therapy prefers a method of stimulating and adjusting the Qi of meridians and collaterals to prevent and treat diseases by applying a micropulse current to the needle after the filiform needle is inserted into the acupoints to get Qi. Previous studies have shown that different acupuncture points, different density, frequency, and intensity of electrical stimulation will bring different therapeutic effects [34]. Electroacupuncture therapy is better than the previous drug treatment in terms of safety and can objectively control the amount of stimulation and stimulate acupoints stably and continuously for a long time [35]. It is cheap and easy. It is more and more widely used and important in clinical work and experimental research [36]. Electroacupuncture reduced NIHSS in individuals with cerebral infarction, according to these findings (mean difference = −2.10, 95% CI: -2.53–-1.67, *p* < 0.00001).

The present study has some limitations. Firstly, all citations only researched that the effects of electroacupuncture presented cerebral infarction. Second, due to a relatively low number of studies included which depicted the relationship between electroacupuncture and the therapy of a stroke in the brain, it is an important reason for the heterogeneity of this results. To corroborate our findings, we would need to conduct high-quality, large-scale investigations with more diverse patient populations. Furthermore, we found significant heterogeneity for multiple factors; nevertheless, we employed a fixed-effect ability to estimate for the heterogeneity, which was also present due to differences in included research.

## Figures and Tables

**Figure 1:** Characteristics of the studies that were included.

**Figure 2:** Characteristics of included studies. Risk of bias summary (a). Risk of bias graph (b).

**Figure 3:** The effects of electroacupuncture on BI, Fugl-Meyer index, CSS, and NIHSS of cerebral infarction: BI (a), Fugl-Meyer index (b), CSS (c), and NIHSS (d) of cerebral infarction.

**Figure 4:** All of the funnel plots were symmetric, suggesting that there was no clear publishing bias: BI (a), Fugl-Meyer index (b), CSS (c), and NIHSS (d) of Publication bias.

**Figure 5:** The mean difference of electroacupuncture on BI, Fugl-Meyer index, CSS, and NIHSS of cerebral infarction.

**Table 1:** Included studies basic characteristics.

Study year	Country	Ethnicity	Cases	Gender (M/F)
Lee et al. 2020	Korea	East Asia	46	22/24
Pei et al. 2001	China	East Asia	86	43/43
Tang et al. 2009	China	East Asia	164	84/80
Xu and Peng 2018	China	East Asia	60	30/30
Zhang et al. 2013	China	East Asia	98	49/49
Zhu et al. 2017	China	East Asia	60	30/30
Wang et al. 2014	China	East Asia	340	170/170

## Data Availability

The data used to support this study are available from the corresponding author upon request.
